# Efficacy of High-Quality Nursing Service for the Patients during the Anesthesia Recovery Period: A Meta-Analysis

**DOI:** 10.1155/2022/3528915

**Published:** 2022-08-08

**Authors:** Hui Li, Heng Wang, Yan Pan, Qian Huang, Xueping Li, Xiaoqi Zeng, Li Zhou

**Affiliations:** Department of Anesthesiology, West China Hospital, Sichuan University, Chengdu 610041, China

## Abstract

**Background:**

To investigate the efficacy of high-quality nursing service for the patients during the anesthesia recovery period.

**Methods:**

We used the National Library of Medicine (PubMed), Cochrane Library of Excerpta Medica Database (EMBASE), China National Knowledge Infrastructure (CNKI), Wanfang, and very important person (VIP) databases for conducting a systematic literature study. We employed the fixed-effects model for evaluating the standardized mean differences (SMDs) with 95% confidence intervals (CIs). The sensitivity and publication bias were estimated for determining the efficacy of high-quality nursing services during the recovery period of anesthesia.

**Results:**

In our study, the result showed that the efficiency of recovery time of spontaneous respiration was significantly improved in the experimental group (SMD = −1.48, 95%CI = [−1.62, −1.34]). In this analysis, the extubation time of the experimental group was lower than that of the control group. In control group [WMD = −15.54, 95% CI (-21.24, -9.83), *P* < 0.00001], the improvement of extubation time was more obvious on high-quality nursing. Moreover, the incidence of agitation in the experimental group was lower than that of the control group, and the score of nursing satisfaction was higher than that in the control group (*P* = 0.01). The funnel plots identified no publication bias during the identification of efficacy.

**Conclusions:**

The high-quality nursing care for patients during the resuscitation period can shorten the recovery time of their self-consciousness and self-breathing, reduce the occurrence rate of restlessness, improve patients' anxiety and depression, reduce complications, and play a certain clinical application effect.

## 1. Introduction

General anesthesia refers to the use of narcotic drugs to enter the patient's body through the respiratory tract, vein, and other channels so that the narcotic drugs can inhibit the central nervous system of the body and make the patient lose consciousness, pain disappear, and unconscious, to achieve the ultimate painless purpose and provide favorable conditions for surgery, medical treatment, and other examinations and treatments [1, 2]. The recovery period of anesthesia refers to the period when the patient stops giving narcotic drugs and waits for the recovery of consciousness of the patient, that is, after stopping narcotic drugs, the patient begins to have pain reaction, become conscious, and recover stable vital signs [3]. During the recovery period of general anesthesia, patients are prone to a series of complications, such as respiratory obstruction, hypoxemia, hypotension, nausea and vomiting, and even ventricular arrest [4]. Therefore, after general anesthesia, the patients need to be closely observed and tested in the postanesthetic care unit (PACU), and the patients cannot be escorted back to the ward until their vital signs are stable, and their consciousness is clear, and their muscle strength is restored.

A mental state in which consciousness and behavior are separated in the recovery period of anesthesia is called “emergence” agitation (EA), which usually occurs about 15 minutes after extubation [5]. It is characterized by excitement, agitation, restlessness, disorientation, and inappropriate behavior, such as unconscious waving of limbs, nonsense, crying, or moaning. Although agitation lasts for a short time and can subside on its own, it increases the risk of patients' self-injury and unplanned extubation, and delayed discharge increases the workload of medical staff and hospitalization expenses of patients and is also the main reason for the decrease of family members' satisfaction with medical staff [6, 7]. The cause and mechanism of restlessness in the convalescent period have not been clearly explained yet, but restlessness may occur in patients of different ages, with an incidence of 10%-23% [8]. In addition, patients are more likely to have anxiety about postoperative pain, and anxiety and pain are related to the incidence of postoperative restlessness. At present, the preventive measures for postoperative restlessness are mostly game intervention, touch nursing, heat preservation intervention, and so on.

Under high-quality nursing, the nursing staff are arranged to adopt different education and guidance methods for different patients and make the patients fully aware of the care. High-quality nursing care which has been defined as nursing care with additional caring facilities and methods including group nursing, whereby several nurses are assigned to 1 particular patient, with combined nursing measures such as nursing plan, nursing philosophy, and nursing quality evaluation and which involves high-quality nursing modes to achieve the expected goals of treatment smoothly and with fewer complications, should be implemented for patients [8, 9]. This study is aimed at demonstrating the efficacy of high-quality nursing service for the patients during the anesthesia recovery period, which will provide opinion and treatment methods for doctors and nurses for caring of patients.

## 2. Materials and Methods

### 2.1. Strategies for Searching

In our study, the retrieval language is limited to Chinese and English, and the latest retrieval time is up to April 2022. The Chinese databases mainly include CNKI, VIP, and Wanfang-related Chinese search engines; English databases mainly include PubMed, EMBASE, Cochrane Library, ScienceDirect, and related English search engines. At the same time, this paper also traces the references of the retrieved literature again, in order to ensure the comprehensiveness of the retrieval. The search strategy included the following terms: ((“high-quality nursing service”) OR (“nursing service”) AND (“anesthesia recovery period” OR “anesthesia recovery”)).

### 2.2. The Inclusion and Exclusion Criteria of Selected Studies

We set the inclusion criteria described below: (a) all research involving nursing service in the anesthesia recovery period; (b) the main outcome measures included patient's status, extubation time, the incidence of adverse reactions, incidence of complications, and improvement of symptom scores; (c) the patients in the treatment group received high-quality nursing during operation, while those in the control group received routine nursing or other nursing measures.

In addition, we set the following exclusion criteria: (a) study of observation; (b) research on animals, (c) documents with poor quality or repetitive research, too little reported information, and unusable; (d) severe mental illness and heart, liver, and other major organ diseases cannot be evaluated.

### 2.3. Quality Assessment of Extracted Data

Both investigators searched independently, analyze, screened, and excluded duplicate kind of literatures and the literature that did not conform to the subject, and paid attention to the unpublished dissertations and conference papers. Preliminary screening will be conducted for crossreview and finally included in the results. And discuss, modify, delete, and incorporate the existing divergent opinions. Jadad quality evaluation scale was used to evaluate the quality of the literature, which was divided into three cases: ① randomization, randomization, 2 points in total, 2 points for the correct random grouping method of the literature, and 1 point for the descriptive random method; ② double-blind method: 2 points for the double-blind method, 2 points for the descriptive double-blind method, and 1 point for the author's narrative double-blind method only; ③ the score of describing the withdrawal of patients from the experiment is 1 point. The score of describing whether there are participants in the experiment is 1 point. Those who are not mentioned will not get a score. Results: low-quality literature scored 0-2, and high-quality literature scored 3-5.

### 2.4. Computational and Statistical Analysis

We employed the Review Manager Software (RevMan, V:5.2) for analyzing the data and outcome indicators in this study. We identified the effect model based on the heterogeneity test results. If *I*^2^ ≥ 50% in the heterogeneity test, we selected the random effect model (RE). In contrast, if *I*^2^ ≤ 50% in the heterogeneity test (within the acceptable range), we selected the fixed-effects model (FE). We combined the continuous variables by applying weighted mean difference (WMD) and combined the binary variables by applying the RR. We considered *P* < 0.05 for significant differences in every outcome index. We utilize the subgroup analysis for identifying the origin of heterogeneity. Moreover, we employed the sensitivity analysis for assessing the influence of each research on the calculated results.

### 2.5. Ethical Statement

This type of secondary analysis or meta-analysis required no ethical consent.

## 3. Results

### 3.1. The Diagrammatic Presentation and Selection of Studies

We detected 296 articles from the Chinese database and English database by using preset measurements and keywords. After software analysis, 125 pieces of literature were excluded, and 171 were left. After reading the full text of the literature, 115 articles that did not meet the inclusion criteria were excluded, and then, further analysis of the literature data was carried out. The flow diagram of the literature search was shown in Figure 1.

### 3.2. Characteristics of Included Studies

The characteristics of included studies are summarized in Table 1. Eight involving high-quality nursing services for the patients during the anesthesia recovery period were included [10–17]. All the experimental groups were treated with high-quality nursing [10–17]. The literature was reported from 1999 to 2021. Meta-analysis identifies the risk of bias in randomized trials included in this study (Figure 2). We performed the randomization based on the computer-aided random list or using a randomly generated pattern of numbers within most of the trials [10–17]. The low risk of incomplete outcome data and selection of outcome reports were utilized to characterize the randomized trials taken in this research. Eight studies [10–17] taken in this research were described with blinding of high-risk contributors and staff and assessing the outcome [10–17]. Furthermore, the randomized trials consider the uncertain risk of other biases. In the end, we found the moderate to the high quality of these researches.

### 3.3. The Meta-Analysis of 8 Selected Researches

The meta-analysis of 8 selected researches in this study [10–17] revealed that the efficiency of recovery time of spontaneous respiration was significantly improved in the experimental group (SMD = −1.48, 95%CI = [−1.62, −1.34]; Figure 3).

In this study, we analyzed the forest plot by applying the meta-analysis of extubation time. The 8 included studies [10–17] identified the outcome of extubation time. We found the 2458 samples in the experimental group and 1862 samples in the control group for further analysis. A powerful method, meta-analysis, identified that extubation time was lower in the experimental group when compared with the control group. In control group [WMD = −15.54, 95% CI (-21.24, -9.83), *P* < 0.00001], the improvement of extubation time was more obvious on high-quality nursing, shown in Figure 4.

Furthermore, the analysis of the forest plot identifies the incidence of agitation and nursing satisfaction. The meta-analysis revealed that the incidence of agitation was significantly lower in the experimental group when compared with the control group (*P* = 0.03) (Figure 5), and the score of nursing satisfaction was higher than that in the control group (*P* = 0.01) (Figure 6).

### 3.4. Analysis of Sensitivity and Publication Bias

Investigation of sensitivity demonstrated that elimination of any one research from our inspection did not destabilize the findings of the pooled analysis (data not shown). Publication bias “is a bias in the published literature, where the publication of research depends on the nature and direction of study results.” In addition, the funnel plots were analyzed for evaluating the bias of publication. We found no publication bias using the efficacy of funnel plots (Figure 7).

## 4. Discussion

The present meta-analysis demonstrated that the efficiency of the recovery time of spontaneous respiration was significantly improved in the experimental group (SMD = −1.48, 95%CI = [−1.62, −1.34]). In this analysis, the extubation time of the experimental group was lower than that of the control group. In control group [WMD = −15.54, 95% CI (-21.24, -9.83), *P* < 0.00001], the improvement of extubation time was more obvious on high-quality nursing. Moreover, the incidence of agitation in the experimental group was lower than that of the control group, and the score of nursing satisfaction was higher than that in the control group (*P* = 0.01). No publication bias was found by using the efficacy of funnel plots.

The anesthesia and resuscitation room is mainly a unit that closely observes and monitors the patients after the anesthesia operation until all the anesthetic drugs in the patients are metabolized, and the patients are fully awake without special circumstances [18]. General anesthesia surgery patients are managed in the anesthesia recovery room, to ensure the life safety of patients in the anesthesia recovery period [18]; (2) it can provide a comfortable and safe resuscitation environment for patients, to shorten their resuscitation time; (3) increase the turnover rate of the operating room, and improve the utilization rate of operating room; (4) save human resources, reduce costs, and reduce patient treatment costs [19]. The traditional nursing measures in the recovery period of anesthesia have been unable to meet the needs of patients [20]. Therefore, clinical research will focus on exploring what kind of safe and effective nursing methods.

The application of high-quality nursing in the anesthesia recovery room has made the anesthesia nurse the best assistant of the anesthesiologist [21]. While improving the workflow, the daily nursing work has changed from passive to active [22, 23]. It is not only necessary to fully understand the condition of each patient but also to fully understand and understand the treatment intention of the anesthesiologist and implement the doctor's orders timely and accurately, enhancing the spirit of unity and cooperation with the anesthesiologist. It ensures the life safety and the best physiological state of patients and acts as a bridge and link between doctors and patients [24–26]. The application of high-quality nursing in the anesthesia recovery room has strengthened the nurses' awareness of active service and responsibility [26, 27]. High-quality service not only improves the quality of nursing staff but also improves patients' satisfaction, avoids disputes and errors, achieves good results, and wins praise from doctors and patients [28].

The study has a few drawbacks. The key drawback is that we take the researches from a limited region. We have taken 21 pieces of research conducted in the eastern. In addition, other factors were considered as a confounder, because our findings in this research were constructed according to the unadjusted estimates. Moreover, we incorporated a lower number of sample-size, single-centric researches with the heterogeneity of clinical aspects, and backgrounds of patients with variable factors, which ultimately lead to a lower level of statistical power and inconsistent findings among the included studies. In the end, the clinical trials using the large sample sizes are necessary to assess the efficacy and safety of pramipexole in Parkinson's disease with anxiety or depression.

## 5. Conclusion

In conclusion, the application of high-quality nursing care in the anesthesia and resuscitation of patients undergoing general anesthesia surgery can reduce the restlessness rate, improve their bad mood, reduce complications, shorten the time of anesthesia and resuscitation, and play a certain clinical effect.

## Figures and Tables

**Figure 1:** Flow diagram of the literature search.

**Figure 2:** The risk of bias was included in the meta-analysis.

**Figure 3:** Efficacy of high-quality nursing on the recovery time of spontaneous respiration. *P* < 0.00001, ^∗∗∗^. With heterogenity 2.86, Chi^2^ = 407.66, df = 7, *I*^2^ = 98%.

**Figure 4:** Efficacy of high-quality nursing on extubation time. *P* < 0.00001, ^∗∗∗^. With heterogenity 67.59, Chi^2^ = 9568.05, df = 7, *I*^2^ = 100.

**Figure 5:** Efficacy of high-quality nursing on the incidence of agitation. *P* = 0.03, ^∗^. With heterogenity 0.09, Chi^2^ = 13.10, df = 5, *I*^2^ = 62%.

**Figure 6:** Efficacy of high-quality nursing on nursing satisfaction. With heterogenity 0.56, Chi^2^ = 36.15, df = 7, *I*^2^ = 81%.

**Figure 7:** The funnel plots for effect were shown.

**Table 1:** Characteristics of the 8 studies in the meta-analysis.

Author year	Country	Size EG/CG	Types of studies	Intervention
Berning 2017 [10]	Switzerland	40/40	Retrospective study	High-quality care/routine care
Dahlberg 2022 [11]	Sweden	217/262	Perspective study	High-quality care/routine care
Öbrink 2019 [12]	Sweden	37/36	Retrospective study	High-quality care/routine care
Boney 2022 [13]	Canada	250/220	Retrospective study	High-quality care/routine care
Ahmed 2014 [14]	California	512/628	RCT analysis	High-quality care/routine care
Grant 2019 [15]	Sweden	50/50	Retrospective study	High-quality care/routine care
Kiekkas 2019 [16]	Greece	1300/598	RCT analysis	High-quality care/routine care
Arun 2021 [17]	Qatar	28/28	RCT analysis	High-quality care/routine care

## Data Availability

The data used to support this study is available from the corresponding author upon request.
